RETRACTED

# Evaluation of Traditional Culture Teaching Efficiency by Course Ideological and Political Integration Lightweight Deep Learning

**DOI:** 10.1155/2022/3917618

**Published:** 2022-06-25

**Authors:** Qingqing Zhong

**Affiliations:** Shaanxi Police College, Foundation Department, Xi'an 710021, Shaanxi, China

## Abstract

With the development of society, China pays more and more attention to cultural education. The teaching method of introducing ideological and political content into cultural teaching plays an important role in improving the overall teaching quality. However, the traditional methods used to evaluate the quality of culture teaching, curriculum ideological, and political teaching have some problems, such as strong subjectivity and unrepresentative results. Firstly, this work analyzes the connotation of curriculum thought and politics. Secondly, a teaching quality evaluation model based on an improved lightweight convolutional neural network (CNN) is proposed, which mainly judges the students' recognition of teachers' content and teaching methods by identifying the students' expressions in the classroom. Finally, the students of a senior high school in Shanghai are selected as the survey object, and the current situation of ideological and political education (IPE) in the school curriculum is preliminarily understood by issuing a questionnaire; experiments are designed to test the performance of the model. The results show that most of the students in the school do not understand the connotation of IPE, and the teachers cannot accurately and deeply teach the relevant ideological and political knowledge to the students. About 73% and 82% of students prefer that teachers can mention life experience and social skills in class. More than 50% of the students are more willing to accept the course ideological and political activities in the form of lectures and competitions. This indirectly shows that the school lacks the above contents in the current course ideological and political teaching, the teaching method is relatively single, and cannot fully mobilize the enthusiasm of students. Further improvement is needed for these problems in the follow-up. The accuracy of expression recognition of this model is more than 2.9% higher than other algorithms, and the improvement effect of the model is remarkable. To sum up, this work fully understands the current teaching situation of the surveyed schools through questionnaire survey, and puts forward corresponding improvement suggestions. The effectiveness of this model is verified by designing experiments, which proves that it is suitable for the research of teaching quality evaluation.

## 1. Introduction

In recent years, the Chinese government has paid more and more attention to education issues, and the proportion of investment in education has been increasing [1]. High school is a very important stage in the growth of students, which has an important impact on students' absorption of knowledge and all-around healthy development [2]. But in the early days, China is dominated by exam-oriented education. Teachers blindly instill cultural knowledge to students in the classroom and do not pay attention to other aspects of knowledge imparting. This will lead to the problem that students are strong in theory and poor in practical experience. Additionally, students' ideas and psychological problems are also ignored, which is not conducive to their physical and mental development [3]. Based on this, “course ideological and political” came into being. It mainly combines ideological and political education (IPE) with cultural education. It introduces ideological and political theories or hot topics related to current affairs while imparting cultural knowledge to students to improve their interest in the classroom and the diversity of teaching modes. This way of learning can fully mobilize students' enthusiasm for learning and promote students' all-around development [4].

RETRACTED

To explore whether a teaching model is effective, it is necessary to use some technical means to evaluate it, such as issuing questionnaires and combining some computer technology. Guo and Yu designed a big data analysis model of college students' English teaching quality to obtain high-precision evaluation results of English teaching quality. The reliability of the established model is verified by experiments: the accuracy of big data analysis and evaluation of the proposed model is 90.22%, which can provide a good reference value for teaching quality evaluation [5]. Lv put forward the design scheme of integrating data mining technology into the course of the ideological and political course teaching evaluation system, as well as the key technologies in the process of system development. After obtaining the evaluation data, the data mining model of teaching quality evaluation is established, and the indexes of teaching quality evaluation are listed [6]. Su et al. in order to make full use of the college English classroom to carry out ideological and political education in the era of big data, proposed a scheme to evaluate the teaching quality of ideological and political courses by using the analytic hierarchy process [7]. Zhang and Meng pointed out that the current effectiveness evaluation model of IPE had caused serious distortion due to poor data processing ability. To solve this problem, they constructed the effectiveness evaluation model of IPE based on in-depth data mining. The clustering method in data mining was used to clean up and preprocess the actual effect of IPE. The experimental results confirmed that the data processing ability of the model was significantly better than that of the existing model [8].

RETRACTED

The above existing research results show that at present, there are many studies on the use of technical means to evaluate the effectiveness of school IPE, but there are few studies on the effectiveness evaluation of the teaching method of integrating ideological and political content into cultural courses. Whether ordinary students recognize teachers' teaching contents and methods in class will be directly reflected in their facial expressions. The introduction of expression recognition technology into teaching is helpful for the objective evaluation of the teaching effect. Based on this, this work creatively proposes a teaching quality evaluation model based on an improved lightweight convolutional neural network (CNN). The model can be used in mobile devices or embedded devices, and then the expression information of students can be collected in real-time by using relevant devices in the classroom to provide an important reference for the evaluation of the effect of traditional culture teaching and curriculum ideological and political teaching. Firstly, this work describes the relevant theories in detail. Secondly, it gives the specific method and process of constructing the model. Finally, a questionnaire is designed to understand the current situation of curriculum IPE in a senior high school in Shanghai, and the effectiveness of this model is verified by designing experiments.

## 2. Materials and Methods

### 2.1. Theoretical Analysis of CIP

In the process of growth, students not only need to absorb more cultural knowledge but also need to establish a correct outlook on life, values, and the world outlook through the correct guidance of parents, teachers, or schools. However, this cannot be effectively achieved by relying only on a certain teacher or individual courses [9]. A student's all-around development of moral character and wisdom requires multiparty cooperation, and the proposal of the “CIP” theory provides a new way to solve these problems [10]. CIP is a kind of educational activity that mainly integrates IPE ideas into the teaching process of various subjects. It can not only teach cultural knowledge but also train students to establish correct concepts and excellent morality, laying a good foundation for students' all-around development [11]. CIP mainly has two characteristics: latent and ideological attributes, as shown in Figure 1.

RETRACTED

In Figure 1, the latent characteristics of CIP mainly mean that IPE is integrated into the teaching process of various disciplines rather than directly imparting relevant ideological and political knowledge to students. By incorporating ideological and political values and concepts into the classroom, this subtle teaching method can alleviate the resistance of students so that students can receive ideological education unconsciously, which is conducive to their healthy development [12]. The characteristics of ideological attributes mainly mean that the ideology of CIP is very clear, which is to guide students to form a firm political position and political persistence so that they can establish correct concepts and eventually have a sound personality. These two characteristics of CIP are indispensable and complement each other. This teaching model combines general education, cultural knowledge transfer, and ideological education, making the teaching mode more diversified. This can fully mobilize students' enthusiasm and provide important support for the comprehensive and healthy development of students [13].

### 2.2. Teaching Quality Evaluation Model Based on Improved Lightweight CNN

Usually, the quality of teaching can be assessed according to students' classroom performance, including their expressions and behaviors. Students' recognition of what and how teachers teach is directly reflected in their facial expressions. Therefore, the introduction of facial expression recognition technology into the teaching process has a certain guiding significance for grasping the actual teaching effect and improving the teaching mode.

#### 2.2.1. CNN

CNN is a typical discriminative deep structure based on minimizing the requirements of preprocessing data. It is one of the representative algorithms of deep learning and is mainly used in research fields, such as computer vision and natural language processing [14]. CNN is mainly built inspired by the structure of human vision and can perform supervised and unsupervised learning. The convolution kernel parameter sharing in the hidden layer and the sparsity of the connection between the layers enable CNN to extract grid-like topology features with a small amount of computation [15]. CNN comprises three parts: convolutional layer, pooling layer, and fully connected layer. Among them, the convolution layer is mainly responsible for extracting the local and global features of the input data, and the pooling layer is responsible for reducing the parameter magnitude. Finally, the underlying parameters are mapped to the new space at the fully connected layer to aggregate the parameters and perform further computations, thereby realizing the fast, efficient, and accurate acquisition of the feature information of the data [16].

RETRACTED

The representation learning ability of CNN enables it to learn the internal features of the data and optimize the model structure and parameter quantity. Usually, the shallower convolutional layers at the front end of CNN can learn local features, such as image texture with a smaller receptive field. The deep convolutional layer at the back end uses a larger receptive field to learn abstract features, such as the size and orientation of objects in the image [17]. The convolution operation is shown in

(1) $$\begin{array}{c} d\left(x,y\right)=\sigma \left(\overset{N-1}{\underset{N=0}{\sum }}\overset{M-1}{\underset{M=0}{\sum }}w^{N,M}u\left(x+n,y+m\right)+b\right), \end{array}$$

where *σ* () represents the activation function; *N* and *M* represent the length and width of the convolution kernel, respectively. *w*^*N*,*M*^ represents the weight of the convolution kernel at the pixel point (*n*, *m*). *u* represents the image feature. *b* represents the offset parameter.

#### 2.2.2. Improvement of CNN

Currently, the most widely used activation function in CNN is rectified linear unit (ReLU). Compared with the traditional sigmoid function, the convergence speed during training has been greatly improved [18]. However, ReLU function is asymmetrical. If the input or weight follows symmetrical distribution, the distribution of the resulting output by this function may be asymmetrical. This will have a certain impact on the actual performance of the network model [19]. Therefore, parametric rectified linear unit (PReLU) function is used instead of ReLU function. PReLU is parameterized ReLU function [20]. The difference between the two is shown in Figure 2.

As Figure 2 indicates, when the input is a positive number, the PReLU function image is consistent with ReLU function, which can avoid the problems of gradient explosion and disappearance. When the input is negative, the gradients of ReLU function will all become 0, while the gradient parameter a_i of PReLU function exists. It can effectively solve the problem of the disappearance of network neurons in the negative region and improve the accuracy of the model [21]. PReLU function is shown in

(2) $$\begin{array}{c} \text{PReLU}=\left\{\begin{array}{cc} x_{i} & x_{i}\geq 0,\\ a_{i}x_{i} & x_{i}<0, \end{array}\right. \end{array}$$

where *x*_*i*_ is the input to the function on the *i*th channel. *a*_*i*_ is the slope coefficient for the negative region. When *a*_*i*_=0, PReLU function is consistent with ReLU function. PReLU can be trained with other layers in the model using the back-propagation algorithm to achieve co-optimization. The updated formula of *a*_*i*_ can be obtained by the chain rule. The *a*_*i*_ gradient of the model layer is shown in

(3) $$\begin{array}{c} \frac{\partial \varepsilon }{\partial a_{i}}=\sum_{x_{i}}\frac{\partial \varepsilon }{\partial f\left(x_{i}\right)}\frac{\partial f\left(x_{i}\right)}{\partial a_{i}}, \end{array}$$

where *ε* is the objective function; *∂ε*/*∂f*(*x*_*i*_) is the gradient propagated from the update layer. The gradient calculation of the activation function is shown in

(4) $$\begin{array}{c} \frac{\partial f\left(x_{i}\right)}{\partial a_{i}}=\left\{\begin{array}{cc} 0 & x_{i}\geq 0,\\ x_{i} & x_{i}<0. \end{array}\right. \end{array}$$

The update of *a*_*i*_ mainly adopts the momentum method, as shown in

(5) $$\begin{array}{c} \Delta a_{i}=\mu \Delta a_{i}+\varepsilon \frac{\partial \varepsilon }{\partial a_{i}}, \end{array}$$

where *μ* is the momentum coefficient. *ε* is the learning rate. Since the learning rate is usually less than 1, PReLU function is usually initialized with *a*_*i*_=0.25.

RETRACTED

#### 2.2.3. Improve the Construction of Lightweight CNN Models

Within a certain range, the depth of CNN is proportional to its accuracy. However, many weight parameters are generally stored in deep CNN. These parameters have high requirements for equipment [22]. Now the devices used for facial expression recognition have gradually shifted to mobile devices and embedded devices. These devices have limited capacity and generally cannot carry deep CNN. The models need to be compressed into lightweight CNN before they can be used. Compressing the model has an impact on its accuracy [23]. The performance of the model needs to be optimized to solve this problem, and the amount of computation needs to be reduced in a certain way.

Based on this, an improved lightweight CNN model is proposed. PReLU function is used in the model, and the model is optimized by stochastic gradient descent. Meanwhile, principal component analysis (PCA) is used to perform dimensionality reduction on the input data. This processing method preserves the main information while removing redundant information, thereby improving the efficiency and accuracy of lightweight CNN.

The essence of stochastic gradient descent is to seek the minimum value of loss function so that the training loss of the model is minimized and the accuracy is the highest [24]. The loss function of the sample is shown in

(6) $$\begin{array}{c} \text{Loss}\left(\theta_{j}\right)=\text{Loss}\left(\theta_{j}\right)+\gamma \left(y_{i}-h\left(x_{i}\right)\right)x_{j}, \end{array}$$

where *γ* is the learning rate. It is a key parameter that controls the update of the weight value, and its value has an important impact on the model accuracy. *y*_*i*_ is the predicted value for a random sample. *h*(*x*_*i*_) is the actual value of the random sample.

RETRACTED

Currently, PCA is one of the most used dimensionality reduction methods. The core of the method is to recombine the data of a group of variables with a certain correlation into a group of new linear unrelated variables through the linear transformation without losing the information conveyed by original indexes to achieve the purpose of characteristic compression explanatory variables. The transformed variables are the principal components [25]. PCA has four steps:

(1) The processed data is arranged into a matrix *X*, as shown in
  (7) $$\begin{array}{c} X=\left[\begin{array}{ccc} x_{11} & \ldots & x_{1n}\\ \vdots & \ddots & \vdots \\ x_{k1} & \ldots & x_{kn} \end{array}\right]=\left[\begin{array}{c} X_{1}\\ \vdots \\ X_{K} \end{array}\right], \end{array}$$
*x*_*kn*_ is the new index value after standardizing the original data; *n* is the number of indicators contained in each data; *k* is the total amount of data; *X*_*K*_ is a vector of data for each row in the matrix.
(2) The covariance matrix Y of the calculation matrix *X* is calculated as shown in
  (8) $$\begin{array}{c} Y=\left[\begin{array}{ccc} y_{11} & \ldots & y_{1k}\\ \vdots & \ddots & \vdots \\ y_{k1} & \ldots & y_{kk} \end{array}\right], \end{array}$$
*Y* is a real symmetric matrix of order *k*, which has *k* real eigenvalues, and the eigenvectors corresponding to different eigenvalues intersect each other.
(3) The eigenvalues of matrix *Y* and their corresponding unit eigenvectors is calculated.
The first *p* eigenvalues are arranged in descending order as the eigenvectors *a*_*p*_ corresponding to *λ*_1_, *λ*_2_,…, *λ*_*p*_, *λ*_*p*_, which is the coefficient set of the obtained principal component index *B*_*m*_ corresponding to the original index vector *A*_*m*_, assuming
  (9) $$\begin{array}{c} a_{p}={\left\{b_{1},b_{2},\ldots ,b_{p}\right\}}^{T}. \end{array}$$
There are
  (10) $$\begin{array}{c} Y_{p}=a_{p}B_{p}. \end{array}$$
The contribution rate *g*_*j*_ of the new comprehensive indicator *B*_*j*_ to the overall variance is shown in
  (11) $$\begin{array}{c} g_{j}=\frac{\text{variance}\left(B_{j}\right)}{\sum_{i=1}^{m}\text{variance}\left(B_{i}\right)}. \end{array}$$
If the contribution rate is high, it means that the principal component contains more information.
(4) The number of principal component indicators is determined.
Usually, the cumulative variance contribution rate *G*(*j*) is used to judge the number of principal component indicators, as shown in equation (12) [26].
  (12) $$\begin{array}{c} G\left(j\right)=\frac{\sum_{i=1}^{j}\lambda_{i}}{\sum_{k=1}^{m}\lambda_{k}}. \end{array}$$

Generally, there are two selection methods. First, when the value of *G*(*j*) is greater than 80%, the value of *j* is the number of selected principal component indicators. Second, we select the unit eigenvector corresponding to the eigenvalue of *λ* > 1 to form a transformation matrix for principal component selection. The number of principal components is the number of eigenvalues that meet the conditions. The main steps of PCA are shown in Figure 3.

RETRACTED

The structure of the constructed improved lightweight CNN model is shown in Figure 4.

In Figure 4, the constructed model has a total of 10 layers. Among them, there are five convolutional layers, one max-pooling layer, one average pooling layer, two fully connected layers, and one output layer. PReLU function is added to each convolutional layer to perform convolution operations on the input image to refine the local features of the image gradually. The pooling layer mainly pools the image to reduce the image dimension and the number of parameters. The fully connected layer mainly integrates the extracted features to ensure the accuracy of the model. The last layer is the Softmax output layer, which mainly classify integrated features and finally get the result. The workflow of the model is shown in Figure 5.

Figure 5 suggests that the model work can be divided into two parts: data initialization and CNN model training. Input the original image dataset, divide the dataset into two parts: training dataset and inspection dataset, and label the expression category of the dataset with index, respectively. After that, extract the principal component feature image of the dataset and enhance the data, which is used for the input of the CNN model.

### 2.3. Questionnaire Design of the Current Situation of CIP Teaching

This work designs an expression recognition model based on improved lightweight CNN to accurately and objectively evaluate the effect of traditional culture teaching and ideological and political teaching. However, the premise of all teaching quality evaluation work is to have a full understanding of the current teaching situation. On this basis, combined with the teaching quality evaluation model proposed here, some improvement strategies can be further put forward, constantly improving the teaching mode and the teaching quality. The method of offline distribution of questionnaires is used to investigate and analyze the current situation of CIP teaching. Students from a high school in Shanghai are selected as the survey subjects. A total of 120 questionnaires are distributed, 118 are recovered, 115 are valid questionnaires, and the effective recovery rate is 95.8%. A total of 7 questions are set for these three dimensions, as shown in Figure 6.

RETRACTED

Figure 6 shows that this survey is mainly divided into three dimensions: first, students' understanding of curriculum thought and politics, corresponding to questions 1 and 2, respectively; second, students' feelings about teachers' teaching ideological and political knowledge correspond to questions 3, 4, and 5, respectively; third, the teaching method expected by students, corresponding to questions 6 and 7, respectively.

### 2.4. Model Testing Experimental Design

#### 2.4.1. Dataset

Three public datasets for expression recognition technology evaluation are used to validate the model's performance, namely the Ck+ dataset [27], the Jaffe dataset [28], and the Fer-2013 dataset [29]. The Ck+ dataset contains 327 video sequences from 123 subjects. Among them, 118 subjects' expressions are marked with anger, contempt, disgust, fear, happiness, sadness, and surprise. The Jaffe dataset contains six basic facial expressions and one neutral facial expression, with a total of 213 static images of size 256 ∗ 256. Each expression in the Jaffe dataset has different expressions derived from different subjects. Therefore, it is challenging for this dataset to be used for experiments. The Fer-2013 dataset is established by intercepting facial expression images from Internet videos, which contains 35,887 48 ∗ 48 gray images and seven types of expression labels. This dataset is by far the lowest and one of the most challenging. The samples of these three datasets are all separated by a ratio of 7 : 3, 70% are used as the training set, and the remaining 30% are used as the test set to validate the model.

#### 2.4.2. Specific Experimental Methods

During the experiment, traditional CNN and improved CNN are used as controls, and the expression recognition accuracy (Accuracy) is used as the indicator. The performance of the proposed improved lightweight CNN model is verified. Accuracy is calculated as

(13) $$\begin{array}{c} \text{Accuracy}=\frac{\left(\sum_{j=1}^{N}n_{jj}\right)}{\left(\sum_{i=1}^{N}\sum_{j=1}^{N}n_{ij}\right)}, \end{array}$$

where *n*_*ij*_ indicates the number of samples whose actual label is *i* and the recognition result is *j*. *n*_*jj*_ is the number of samples whose actual label and recognition result are both *j*. *N* represents the total number of samples. The larger the value of Accuracy, the better the expression recognition performance of the model.

The setting of the learning rate parameter has a great influence on the accuracy of the model. Therefore, before carrying out the formal experiment, the Jaffe data set shall prevail, and the learning rate of the model shall be optimized. The learning rate range is set to (0.001 and 0.002). The maximum number of training sessions is 400.

RETRACTED

## 3. Results and Discussion

### 3.1. Survey Results of the Current Situation of CIP Teaching

  Dimension 1: the survey results of students' understanding of CIP are shown in Figure 7.
  In Figure 7, only 10.43 of the students really knew about CIP, and less than 10% of the students knew the difference between CIP and ideological and political courses. It shows that most high school students in this region have no in-depth understanding of the current education form and purpose and lack of concern for the country's education policy, which is not conducive to the development of the CIP teaching model. Therefore, teachers should be good guides in the classroom, leading students to fully understand the connotation and importance of CIP to gradually adapt to the new teaching mode and lay a solid foundation for the all-around development of students.
  Dimension 2: the results of the survey on students' feelings about teachers' teaching of ideological and political knowledge are shown in Figure 8.
  In Figure 8, some teachers of the school will explain ideological and political knowledge and current hot topics in the classroom. A small number of students also gave certain affirmations to CIP. However, most teachers do not explain these contents clearly, so the teaching effect is very limited. Schools should strengthen the training of teachers in various disciplines in the later stage so that they can fully understand ideological and political knowledge and accurately convey it to students.
  Dimension 3: the results of the survey on the teaching style that students expect are shown in Figure 9.
  In Figure 9, students not only want to learn cultural knowledge but also hope that teachers can teach knowledge about entertainment news, life skills, life, and learning experience in the classroom. This shows that students also want to make their own knowledge base more extensive and comprehensive. Additionally, students are more willing to accept CIP activities in the form of lectures and competitions. The survey results reflect that the current teachers' teaching methods in the classroom are relatively monotonous, lacking in imparting knowledge of news and life experience, and fail to arouse the enthusiasm of students by organizing related activities. Therefore, these aspects need to be further strengthened.

### 3.2. Model Training and Parameter Optimization Results

#### 3.2.1. Model Training Results

The training results of the proposed improved lightweight CNN model on three datasets are shown in Figure 10.

RETRACTED

In Figure 10, when the model is trained on the Ck+ dataset, the recognition accuracy of the expressions in the dataset reaches the highest, i.e., 86%, when the number of training times is 80. When training on the Jaffe dataset, the recognition accuracy reached the highest, i.e., 83%, when the number of pieces of training is 90. When training on the Fer-2013 dataset, due to the large and complex dataset, the recognition accuracy reached the highest, i.e., 78%, only when the number of pieces of training is 110 times. In general, the training speed of the model is faster, the accuracy is higher, and the performance is better.

#### 3.2.2. Optimization of Model Learning Rate Parameters

When different learning rate values are set, the expression recognition accuracy of the proposed improved lightweight CNN model on the three datasets is shown in Figure 11.

In Figure 11, the learning rate is mainly used to control the updated speed of the parameters when the model is trained, and the selection of its value has an important impact on the performance of the neural network. When the learning rate is too large, the parameters will fluctuate around the minimum value and cannot approach the optimal solution. When the learning rate is too low, the number of iterations of the model will increase, the amount of calculation is large, and the phenomenon of overfitting is prone to occur. When the learning rate is 0.0014, the expression recognition accuracy of the model reaches the maximum. Therefore, the learning rate of the model is set to 0.0014.

### 3.3. Model Performance Test Results

With traditional CNN, improved CNN, and the improved lightweight CNN model, the expression recognition accuracy on the three datasets are shown in Figure 12.

In Figure 12, according to the overall curve trend, the models on the three datasets have the highest accuracy for expression recognition. The average recognition accuracy of traditional CNN is 81.28%. The average recognition accuracy of improved CNN is 82.76%. The average recognition accuracy of the models is 85.17%.

To sum up, the average accuracy of expression recognition of the proposed improved lightweight CNN model on the Ck+ dataset, the Jaffe dataset, and the Fer-2013 dataset is higher than traditional CNN and improved CNN by 4.8% and 2.9%, respectively. The model improvement effect is remarkable. Therefore, the model is suitable for recognizing students' expressions in the classroom. Based on the recognition results, it is possible to clarify the students' recognition of the teaching content and teaching methods to evaluate the effectiveness of the CIP teaching model.

RETRACTED

## 4. Conclusion

In the past, teaching quality evaluation is mainly conducted by employing questionnaires, which is highly subjective. A teaching quality evaluation model based on an improved lightweight CNN model is proposed to evaluate the teaching effect through student expression recognition. A preliminary understanding of the current situation of CIP education in a high school in Shanghai is conducted by issuing questionnaires, and an experiment is designed to test the performance of the model. The results show that the school's CIP education work needs further improvement. Teachers' mastery of the ideological and political theory is insufficient. Students do not know enough about the connotation of CIP. Teachers' teaching methods are relatively simple and cannot fully mobilize students' enthusiasm. The model's recognition accuracy for expressions is 4.8% and 2.9% higher than traditional CNN and improved CNN, respectively. The model improvement effect is significant. However, this work only uses the existing public dataset to verify the performance of the model, which needs to be introduced into the classroom for field research in the future. These results can provide an important reference for evaluating traditional culture teaching and the CIP teaching effect.

## Figures and Tables

**Figure 1:** Features of CIP.

**Figure 2:** ReLU function: (a) ReLU function; (b) PReLU function.

**Figure 3:** Main steps of PCA.

**Figure 4:** The structure of the improved lightweight CNN model.

**Figure 5:** Workflow for improving a lightweight CNN model.

**Figure 6:** Specific content of the questionnaire.

**Figure 7:** Survey results of students' understanding of CIP ((a) survey results of questionnaire item 1; (b) survey results of questionnaire item 2).

**Figure 8:** Survey results of students' feelings about teachers' teaching of ideological and political knowledge: (a) survey results of questionnaire item 3; (b) survey results of questionnaire item 4; (c) survey results of questionnaire item 5.

**Figure 9:** Survey results of students' expectations of teaching methods: (a) survey results of questionnaire item 6; (b) survey results of questionnaire item 7.

**Figure 10:** The training results of the model: (a) the training results on the Ck+ dataset; (b) the training results on the Jaffe dataset; (c) the training results on the fFer-2013 dataset.

**Figure 11:** The recognition accuracy of the model under different learning rates.

**Figure 12:** Expression recognition performance comparison of the three models.

## Data Availability

The data used to support the findings of this study are available from the corresponding author upon request.
